The article "Presented a Framework of Computational Modeling to Identify the Patient Admission Scheduling Problem in the Healthcare System" was published in 2022. Journal: J Healthc Eng.

# Presented a Framework of Computational Modeling to Identify the Patient Admission Scheduling Problem in the Healthcare System

**DOI:** 10.1155/2022/1938719

**Published:** 2022-11-29

**Authors:** Reza Hosseini Rad, Sahba Baniasadi, Parisa Yousefi, Hakimeh Morabbi Heravi, Muzhir Shaban Al-Ani, Mohsen Asghari Ilani

**Affiliations:** ^1^Department of Industrial Engineering, Amirkabir University of Technology, Tehran, Iran; ^2^Master of Industrial Engineering, Department of Industrial Engineering, University of Houston, Houston, TX, USA; ^3^Department of Industrial Engineering, Qazvin Islamic Azad University (QIAU), Qazvin, Iran; ^4^Department of Statistics, University of Bojnord, Bojnord, Iran; ^5^University of Human Development, College of Science and Technology, Department of Information Technology, Sulaymaniyah, KRG, Iraq; ^6^School of Mechanical Engineering, College of Engineering, University of Tehran, Tehran, Iran

## Abstract

Operating room scheduling is a prominent study topic due to its complexity and significance. The increasing number of technical operating room scheduling articles produced each year calls for another evaluation of the literature to enable academics to respond to new trends more quickly. The mathematical application of a model for the patient admission scheduling issue with stochastic arrivals and departures is the subject of this study. The approach for applying our model to real-world issues is discussed here. We present a solution technique for efficient computing, a numerical model analysis, and examples to demonstrate the methodology. This study looked at the challenge of assigning procedures to operate rooms in the face of ambiguity regarding surgery length and the arrival of emergency patients based on a flexible policy (capacity reservation). We demonstrate that the proposed methods derived from deterministic models are inadequate compared to the answers produced from our stochastic model using simple numerical examples. We also use heuristics to estimate the objective function to build more complicated numerical examples for large-scale issues, demonstrating that our methodology can be applied quickly to real-world situations that often include big information sets.

## 1. Introduction

Patients seeking medical treatment often turn to outpatient services, and their efficiency is critical to patient satisfaction with the healthcare system. Outpatient service operations management has faced a number of challenges in response to the growing demand for outpatient services and the changing behavioral patterns of patients. In today's healthcare system, it is widely recognized that timely and straightforward access to healthcare services must be provided to all patients. In general, there has been an increase in the demand for healthcare services over the past decade. The reasons for this include an aging population and increasing awareness of the benefits of preventative care. In contrast, the global economic crisis is forcing healthcare systems to reorganize. There is a reduction in public healthcare providers at the macro level [1]. Patients can easily access clinics through a good scheduling system [2]. Thus, long patient wait times are caused by inefficient or poorly planned schedules. As a result, there are more complaints and unhappy patients. By recognizing and appreciating the importance of effective patient scheduling, as highlighted by Suss et al., outpatient clinics can use various scheduling strategies to strike a balance between patient satisfaction and resource utilization [3].

The article "Presented a Framework of Computational Modeling to Identify the Patient Admission Scheduling Problem in the Healthcare System" was published in 2022. Journal: J Healthc Eng.

Furthermore, outpatient clinics' use of appointment systems was praised by patients as a sign of competent service delivery [4]. Consumers perceive that scheduling appointments enhances patient accessibility and satisfaction in a significant way [4]. A study by Sprentrup et al. concluded that appointment systems' dependability, particularly in clinics, had been widely acknowledged as a means to ensure improved patient care and organizational incentives [5, 6]. The most popular methods of scheduling in healthcare are walk-ins and appointments [6–10]. Walk-in scheduling techniques are popular because they are able to maintain a continuous patient flow. According to this method, patients are treated based on a first-come, first-served basis [11]. The appointment system is unique, in that it includes certain delimited intervals or slots in a schedule that can accommodate patients on the same day they seek or apply for an appointment. Schoenfelder et al. concluded that each scheduling approach aims to improve one metric at the expense of another. Therefore, it may be difficult to achieve a balance between patient contentment and resource utilization using a single scheduling strategy [12]. Two scheduling strategies are used by HAS to increase its ability to meet both patient and clinic needs. While appointments allow patients to shorten wait times, walk-ins allow them to enter the facility without an appointment, giving them more freedom [6]. As well as reviewing numerous papers written in English and published in peer-reviewed journals, we searched databases covering a variety of disciplines, such as Scopus and Google Scholar, for relevant articles using terms such as “nurse scheduling,” “nurse rostering,” “patient admission scheduling,” “patient to bed assignment,” “operating room scheduling,” and “operating theater scheduling.” We conducted a forward and backward search for the publications identified to identify related papers. We only examined English-language articles published between 2010 and 2020 (see Figure 1). All articles describing the implications of metaheuristics in arranging healthcare decision-making within an optimization setting were also considered.

The article "Presented a Framework of Computational Modeling to Identify the Patient Admission Scheduling Problem in the Healthcare System" was published in 2022. Journal: J Healthc Eng.

The scheduling of patients is the subject of several studies since it affects the length of time it takes for patients to be seen, as well as the waiting time and idle time in the system over time. Outpatient clinics employ single queues, according to Brahimi and Worthington. Depending on their arrival time, patients may have to wait in long lines. However, such a strategy is ineffective since patients' needs differ. According to Brahimi and Worthington, some people may come to the center for non-health-related consultations, but others may need immediate medical care. In order to ensure increased operating efficiency, a more efficient scheduling approach is required. In addition, each patient is assigned a specific period of time; therefore, the time slot may be squandered if a customer fails to show up. Nevertheless, Aburayya et al. noted that the health center loses money [3].  Section 2 examines the current literature on outpatient scheduling difficulties. In Section 3, we discuss essential patient planning programs by implementing flow and model thinking to better understand general service time distribution and overall performance criteria of current appointment scheduling methods.  Section 4 discusses a number of healthcare application areas and methodologies. The patients' choice function, on the other hand, covers a wider range of topics. Provider selection impacts carrier fines and healthcare income, day of the week selection impacts carrier delays, and appointment time selection impacts patient convenience.  Section 5 concludes with a discussion of the results and recommendations for the future. The mathematical application of a model for the patient admission scheduling issue with stochastic arrivals and departures is the subject of this study. The approach for applying our model to real-world issues is discussed here. We present a solution technique for efficient computing, a numerical model analysis, and examples to demonstrate the methodology. This study looked at the challenge of assigning procedures to operate rooms in the face of ambiguity regarding surgery length and the arrival of emergency patients based on a flexible policy (capacity reservation).

## 2. Previous Investigations

The goal of this review, as stated before, is to examine outpatient appointment scheduling approaches and compare different tactics to explain the benefits of appointment scheduling. Over the last few decades, outpatient appointment scheduling has piqued the interest of various academics and clinicians, starting with the work of Welch and Bailey [13]. In recent decades, the literature has properly covered appointment scheduling, including outpatient scheduling [14], operation room scheduling [15–24], and medical examination scheduling [25–29]. The primary issues with appointment scheduling are connected to optimizing healthcare resources through better usage of human resources and medical equipment, which results in shorter patient wait times. Numerous research studies have found that patient dissatisfaction with outpatient scheduling is typically due to long wait times and that reasonable wait times are necessarily based on clinical competency [30]. Simulation models are among the most well-known methods for examining the impact of random variables on patient wait times and idle doctor time in appointment scheduling [31]. For the issue of appointment scheduling, Granja et al. [32] presented a simulation model optimization method. The suggested simulation model demonstrates good effectiveness in the assessment of medical imaging processes. The patient appointment scheduling is optimized using a simulated annealing approach, which reduces the average service period and overall patient waiting times.

The article "Presented a Framework of Computational Modeling to Identify the Patient Admission Scheduling Problem in the Healthcare System" was published in 2022. Journal: J Healthc Eng.

In comparison to the existing scenario, the whole service time and patient waiting time have been decreased by roughly 5% and 38%, respectively, according to the acquired results. Zonderland et al. [1] investigated an open-access policy that expanded a system and suggested an appropriate heuristic policy for patient-cancelable appointment scheduling. They showed a model that takes data from a real clinic and examines it section by section using a heuristics approach. With all of the other measures in place, many patients have above-average performance. According to Zhao et al. [33], there is a growing trend toward web-based appointment systems. They discussed the benefits of a wide range of patient outcomes from web-based scheduling that overlapped with other research. Early patient acceptance and continued use of a conventional appointment scheduling system were studied by Grain [34]; however, the usual kind of customer utilized an E-Health Service and an E-Appointment Scheduling system. The study was based on a review evaluation to gather relevant information from patients, such as their approval of the system, their thoughts on its features, and their justifications for utilizing it.

Wu et al. [35] devised scheduling principles that define a succession of review responsibilities and different services. The simulation findings assign functions to correct the service time, support the pharmaceutical task across many resources, and optimize the utilization flow. According to Harding and Bottrell [36], waiting times for outpatient physiotherapy were percent shorter in the year after implementing the triage model's specified, timely appointments [33, 34]. Rohleder and Klassen [37] presented a framework for distinguishing patients' viewpoints, reducing the number of times doctors are idle and the number of times patients are waiting. Kong et al. [38] created a robust distributional model that reduces the total cost of patient waiting time. They also provided a model that considered a service provider's idle and overtime to optimize patient arrival times. This approach is challenging because calculating the total cost of a schedule requires linear integer programming with uncertainty in both the goal characteristic and the structure of the restrictions. A new perturbation approach was developed by Liu et al. [39] to improve the dynamical stability of digital chaotic maps. Wu et al. [40] proposed a distributed architecture to permit the scalability of several association-rule-based recommendation algorithms. Wu et al. [41] studied an efficient SQL-to-MapReduce Translator (CAT) that is cost-aware. CAT stands out for two reasons. Based on digital footprint images, Sharifi et al. [42] proposed a new method to diagnose tired feet. Abadi et al. [46] combined the salp swarm algorithm with genetic algorithms to develop a novel method for scheduling nurses for the care of COVID-19 patients. Eslami et al. [44] investigated an attention-based multiscale convolutional neural network (A+MCNN) for automatically classifying frequent distress and non-distress items in pavement photographs. Zheng et al. [45] compared six state-of-the-art class rebalancing approaches against five common classification algorithms for SBR prediction. They outline eight key conclusions from their empirical investigations, which may be used to advise practitioners in selecting optimal class rebalancing strategies and classifiers for SBR prediction. In a multistage outpatient healthcare system, Diamant et al. [46] developed a unique appointment technique for assessing existing healthcare service deployments and observations. The clinic develops a unique appointment scheduling technique in which patients are assigned to a particular appointment day. However, the absence of decision-making in patients' judgments renders this technique ineffective; therefore, they attempted to overcome this restriction. They used a discrete-event simulation to compare their solutions to heuristic scheduling techniques and assess the quality of their solutions based on structural results. Chervenak et al. [47] suggested investigating the detrimental effects of malignant religion and nationalism on patients' biopsychosocial health and medical professionalism. Davoudi et al. [48] used machine learning to investigate the influence of statins taken before infection on the severe decrease of COVID-19. Jia et al. [49] investigated a probabilistic method to schedule port vehicles. Yazdani et al. [50] suggest an application of eXtended Classifier Systems (XCS) for detecting database intrusions in this research. Rezaei et al. [51] suggested a data-driven technique for segmenting the hand parts on depth maps that does not need any additional work to produce segmentation labels. The proposed technique learns to predict the hand form and posture given a depth map by using the labels previously supplied by public datasets in terms of main 3D hand joint positions. Sadeghipour et al. [52] suggested an Intelligent Diabetes Diagnosis System using the XCSLA System. Ahmadi et al. [53] showed how to segment brain tumors using the FWNNet approach. The authors introduced a unique supervised segmentation approach based on the FWNNet layer in this article. Garaix et al. [54] used previously published research to create models that optimize the number of patient visits, reduce affected patient waiting time, and improve patient satisfaction.

The article "Presented a Framework of Computational Modeling to Identify the Patient Admission Scheduling Problem in the Healthcare System" was published in 2022. Journal: J Healthc Eng.

The majority of the literature review studies such as Deng et al. [55] Moreover, Robinson and Chen focused on static modeling techniques [56]. As you can see, the quantity of recent articles has outgrown its capacity.  Figure 2 depicts the proportion of application areas related to patient and outpatient scheduling issues. The majority of extant patient scheduling applications, as can be shown, are in the fields of chemotherapy and radiation. As a result, we suggest a pie chart depicting the many healthcare branches responsible for green outpatient scheduling inside a radiation department, which is defined in such a way as to illustrate various real-life scenarios. The success of the research presented is assessed using haphazardly created problems and a real-life scenario. The results are highly encouraging because the created optimization models enable us to outperform human specialists (see Figure 2).

As seen in Figures 2 and 3, many literature review topics have covered appointment scheduling. In general, the issues are based on highly aggregated data collected at various periods throughout the year. It is worth noting that over half of the contributions are from 2013 or later, demonstrating the growing number of subjects for researchers in the appointment scheduling program. We limit manuscripts to those submitted in or after 2014 and 2015 due to many submissions. Between 2014 and 2015, there were just a few publications published in English on this topic. Nevertheless, due to the collaboration between researchers and the healthcare industry, the number of articles published after 2015 has increased. They recognized that they might profit from the benefits of this approach, such as increased staff productivity and appropriate follow-up for typical chronic disease patients.

The article "Presented a Framework of Computational Modeling to Identify the Patient Admission Scheduling Problem in the Healthcare System" was published in 2022. Journal: J Healthc Eng.

This contribution has enabled scholars in this field to pursue more exciting and new subjects. We have provided a taxonomy of outpatient scheduling concepts and methodologies in. The majority of the research, as described in Appendix, focuses on the modeling techniques discussed previously in this review article, which explored achieving equilibrium between patient waiting time and doctor usage through hospital consultation and resources. In actuality, one of the first practical variables in appointment scheduling is direct and indirect waiting time. Nevertheless, modeling a process indirectly is challenging for a variety of reasons. To begin with, unlike the direct waiting period during which the appointment is terminated, waiting-time difficulties are more accurately depicted as infinite problems. Second, in a schedule conflict, outpatients are given a good appointment time to choose among multiple preferred physicians. ASPs created on a given day for a specific doctor are also linked to various days and physicians.

### 2.1. Decision Level in Production Control

Production planning was defined by Szander et al. [25] and improved by Stamps et al. [26]. The five hierarchical phases of resource capacity management as proposed by Vissers et al. are strategy development, patient volume planning and control, resource planning and control, patient group planning and control, and patient planning and control. Each hierarchical tier is listed below:

Level I: Strategic planning: This is the most high level of the framework. This level of decision-making takes place every two to five years. In addition to being connected to the provider's top executives, they help determine the future direction of the provider.

Level 2: Plan and manage the patient volume: Each patient group has a target number of patients, service levels, and production volume. The process could take up to two years.

Level 3: Resource allocation and control: This section deals with the allocation of resources to groups of patients, such as specialties or departments. These rules determine how patients are grouped. The effects of these activities last from three months to one year.

The article "Presented a Framework of Computational Modeling to Identify the Patient Admission Scheduling Problem in the Healthcare System" was published in 2022. Journal: J Healthc Eng.

Level 4: Patient group planning and control: We are referring to the resources required to perform the patient planning and control function. It takes between three weeks and three months for decisions to be made at this stage.

Level 5: Patient planning and control: This is the area where you arrange daily tasks relating to patient planning. The choices last between one and seven days and relate to the point at which waiting patients are approved. They determine when they will be admitted and released.

Although this approach views healthcare providers as self-contained commercial organizations, it only addresses resource capacity management and ignores online decision-making.

### 2.2. Optimizing Operating Room Scheduling

The scheduling operating room literature has a variety of techniques that apply to the optimization sector. To solve the challenge of operating room scheduling, several heuristics and metaheuristics have been used. [1] Constructing a weekly operating theater operation schedule utilizing an open scheduling method is proposed in this context. This project aims to maximize operating room utilization, reduce operating theater overtime costs, and reduce unplanned idle time among surgical patients. The solution process in this work is divided into two parts. The first step is assigning a particular date for each surgeon to each patient, and surgeons are allowed to allocate their cases to any time block. Then, the daily timetable is established to maintain the operation sequence, taking into account the available recuperation beds. A set-partitioning integer-programming paradigm is used in the suggested technique, and the solution is found via a column-generation-based heuristic procedure. The daily scheduling problem is addressed in the second phase, represented by a two-staged hybrid flow-shop model that is addressed by a hybrid genetic algorithm that employs a Tabu search technique for local search. Depending on Belgian university hospital data, the suggested approach was evaluated with several actual surgical schedules. The findings indicate that there was reduced idle time between surgical patients as a result of the operation schedules as well as more operating room utilization with little overtime. Additionally, [20] created a unique two-stage stochastic mixed-integer-programming approach to handle surgical schedules across many operating rooms under uncertainty. The major point of this study is that the availability of several operating rooms and assistance and support from other surgeons, particularly the chief staff surgeon, allows many procedures to be done concurrently. It explained why surgeons should pool their resources and share them. The following diagram depicts the summary of all optimization algorithms and data collections with categorization (see Table 1).

The article "Presented a Framework of Computational Modeling to Identify the Patient Admission Scheduling Problem in the Healthcare System" was published in 2022. Journal: J Healthc Eng.

## 3. Methodologies

### 3.1. Overlapping Appointment Scheduling Methods

Generally, there are several approaches used in the field of healthcare study. Using appointment scheduling is one of the essential aspects. In this part, various approaches are compared to see one is more practical than the others, using their benefits as a foundation. Just the online or phone services initiate the admission procedure, which may be done with or without an appointment. The primary objective is to reduce access time by allocating specific resources to patients who phone in for an appointment the same day or within a few days [69]. A standard appointment scheduling process for a multidoctor outpatient unit may be reduced to gathering many discrete single-doctor problems [70]. In an outpatient healthcare hospital with a random service time, the overlapping appointment scheduling (OLAS) method minimizes patient awaiting time and doctor idle time while increasing doctor productivity and patient contentment [71]. The OLAS method is used to determine the best overlapping intervals between patient appointments and service hours. Given the probability distributions for patient flow and service time, OLAS is generally framed as an optimization process to reduce the overall cost of patients awaiting and idle doctor time [71, 72]. Much research has been performed to organize patient care time in hospitals utilizing innovative OLAS model techniques. It may be employed to look at a queuing system for patient satisfaction in a hospital setting in a particular field study. Patient satisfaction is essential to any hospital's performance and the public's perception of the hospital as they stand in line for their opportunity to visit a doctor and during their time with the doctor [70]. This finding should aid in the improvement of clinic services and the assurance of the quality of service. Patients' satisfaction with the quality of treatments in outpatient clinics was examined in another research at Egypt's University Hospital, indicating that the healthcare environment requires continuous quality development and attention, notably to please patients [73].

The Monte Carlo (MC) numerical solution may be used to evaluate the findings of optimal overlapping periods provided by an OLAS model as an alternate technique. The OLAS approach may also be employed to test the elements that influence the procedure of establishing an overlap period in clinics, such as service time distribution, over time, and no-shows [74]. The development of an overlap period in clinics with various assumptions is linked to service time distribution over time and no-shows [75]. The lack of particular scheduling services, such as alerts and warnings of overlapping periods, is one of OLAS's significant benefits for appointment scheduling. Despite the cost of extra employees, OLAS enhances overall productivity and profit. In addition, specific appointment analyses place a premium on the number of operation studies. Furthermore, we can expand the MC simulation feature to figure out the number of patients to schedule an appointment with at the start of the session and the duration of a gap between the remaining appointment times using a simulation approach like MC. After this is known, the value may be noted; utilizing this results in a suitable equilibrium between the patient's waiting time and the doctor's idle time. It was observed that the shorter the mean consulting times, the faster the patient's waiting time, and the doctor's idle time decreased [76].

The article "Presented a Framework of Computational Modeling to Identify the Patient Admission Scheduling Problem in the Healthcare System" was published in 2022. Journal: J Healthc Eng.

### 3.2. Model Assumptions

The goal of the MC simulation is to evaluate randomness to provide more accurate findings based on the patient's historical data. MC simulation provides the decision-maker with a variety of probable outcomes and the probability associated with each option. Table 1 categorizes the simulation techniques for outpatient scheduling difficulties. In the simplest optimization model, one customer is included in all modeling to determine the start time of each engaged patient where the OLAS model is particular. For each patient and service level, there are also stochastic factors. For the version, the notation explanation is as follows:

 
*t*_*i*_^*OLAS*^: The appointment begins at the time of patient *i* (OLAS + doctor and patient) for *i* = 1, 2,…, N. *t*_*j*_^*doc*^ The appointment begins at the appointed time for patient *j* (doctor just patient) for *j* = 1, 2,…, *M*.
 
*S*_*i*_^*OLAS*^: OLAS provides service *i* to patients at a set time.
 
*W*_*i*_^*OLAS*^: Patient i's OLAS waiting time.
 
*I*_*k*_: Doctor's idle time between patients *k* and k-1, where *k* = 1, 2,…, *N* + *M.*
  T: Clinic closure time.
  O: The clinic's extra time working. *C*_*w*_^*OLAS*^: The cost of the patients who are waiting for the OLAS.
 
*c*_*w*_^*doc*^: The cost of the patient's time spent waiting for the doctor.
 
*A*_*k*_: Arrival time for the kth patient in the second and A(*k*) is the kth order statistic for *k* = 1, 2,…, *N* + *M.*
 
*W*_*k*_: The time it takes for a doctor to see the kth patient, where W(*k*) is the kth-order statistic for *k* = 1, 2, ..., *N* + *M*.
 
*S*_*k*_: Kth patient visited by the doctor's appointment time, where S(*k*) is the kth-order statistics for *k* = 1, 2, ......, *N* + *M*.

The article "Presented a Framework of Computational Modeling to Identify the Patient Admission Scheduling Problem in the Healthcare System" was published in 2022. Journal: J Healthc Eng.

The definitions that apply are as follows:

(1) $$\begin{array}{c} W_{1}^{\text{OLAS}}=0,\\ W_{i}^{\text{OLAS}}=\max\left\{W_{i-1}^{\text{OLAS}}+S_{i-1}^{\text{OLAS}}-t_{i},0\right\}\text{for}i=2,\ldots \ldots ,N,\\ W1=0\text{ for}k=1,\\ Wk=\max\left\{Wk-1+Sk-1-Ak-1,0\right\}\text{for}k=2,\ldots \ldots ,N+M,\\ I1=0,\\ Ik=\max\left\{Ak-\left(Ak-1+Wk-1+Sk-1\right),0\right\}\text{for}k=2\ldots \ldots ,N+M,\\ O=\max\left\{Ak–\left(Ak-1+Wk-1+Sk-1\;\right),0\right\}–T\text{for}k=N+M. \end{array}$$

Flow time of outpatient

(2) $$\begin{array}{c} i=W_{i}^{\text{OLAS}}+W_{k}+S_{i}^{\text{OLAS}}+S_{k}. \end{array}$$

The goal of the equation is to construct an approximation timetable that minimizes the following function: total projected cost of patient wait length and service point, doctor idle time, and clinic overtime.

We can suppose that *E* follows a uniform distribution in the case of OLAS. Outpatients are anticipated to arrive at different times *t*_1_, *t*_2_,…..*t*_*N*_ and *t*_1_, *t*_2_,……*t*_*M*_ if they come up.

(3) $$\begin{array}{c} {\text{Minc}}_{w}^{\text{OLAS}}E\left[\sum_{i=1}^{n}W_{i}^{\text{OLAS}}\right]+c_{w}^{\text{doc}}E\left[\sum_{j=1}^{m}W_{k}\right]+cIE\left[\sum_{k=1}^{k}I_{k}\right]+\text{co}\left[o\right]. \end{array}$$

*t*_*i*_, *t*_*j*_ subject to

(4) $$\begin{array}{c} t_{1}\geq 0,\\ t_{N}\leq T,\\ t_{1}^{\text{OLAS}}\leq t_{2}^{\text{OLAS}}\leq \ldots \leq t_{N}^{\text{OLAS}},\\ t_{1}^{\text{doc}}\leq t_{2}^{\text{doc}}\leq \ldots \leq t_{M}^{\text{doc}},\\ t_{i},\;t_{j}\mathrm{int}\text{eger.} \end{array}$$

Given that integer values are appointment start instances, it is still accurate that the doctor's maximal work is comparable to *T* − ∑_*J*_*I*_*j*_ +*O* depending on the stated mathematic equations. Outpatients could be accepted earlier, late, or on time for their planned appointment. The OLAS is used to see patients. The doctor line is organized depending on their first appointment time and examination room availability. Patients are displayed in the line according to a first-come-first-served principle. An OLAS-afflicted patient, for instance, can immediately enter the physicians' queue when the OLAS is done.

If a physician-only patient with a later appointment comes before the OLAS, the health doctor will see them first. If there is a vacant examination room, a doctor-only patient will instantly join the medical doctor line. After admittance, all patients are put in exam room lines. A qualified patient is allocated to an exam room if one is accessible or waiting in line. They are in both the OLAS and doctor queues at the same time. As a result of the first appointment and examination room, the number of exam rooms is restricted. Generally, OLAS individuals in an examination room will seek medical assistance sooner than doctor-only individuals who have not yet been allocated a room. Simultaneously, with several phases, overall service examples are generally more significant. The goal is to devise schedules that reduce the accessible ready time for patients while minimizing idle time and time spent outside of the fitness care facility's control. Most OLAS modeling techniques are created for an outpatient healthcare program, and several parameter pairs are mathematically tested. The findings also touch on the topic of appointment scheduling. This approach examines some variables including service time, coefficient, variance, cost ratio, total doctor idle time and overtime, and patient waiting time. Furthermore, numerical studies show that the OLAS approach can considerably cut clinic costs. Outpatients with a long service duration, a high coefficient of variation for service time, a high-cost ratio, and a high no-show rate have the most extended overlap period and lowest cost. As a result, this technique may be studied and contrasted with other appointment scheduling strategies [64].

The article "Presented a Framework of Computational Modeling to Identify the Patient Admission Scheduling Problem in the Healthcare System" was published in 2022. Journal: J Healthc Eng.

Furthermore, discrete-event modeling is a flexible technique designed to form the techniques necessary to alert healthcare scheduling, thanks to those simulation methods types. It provides for a wider range of tools than the Markov standard approach and the creation of procedures at a level appropriate for the task. Its risks are low and easily handled, putting our field closer to the need for strong modes that decision-makers can rely on. To manage the clock in most discrete-event simulations, AnyLogic or Arena Simulation software is used.

### 3.3. Multiple Objectives

Preoperative holding units (PHUs), multiple ORs, postanesthesia care units (PACUs), and intensive care units (ICUs) are the three components of an operating room. They are all useful in supplying effective planning and scheduling for surgical procedures. The most efficient components of the operating room, such as numerous ORs and critical care units, are evaluated in this study's operation schedule (ICUs). Other areas, on the other hand, are believed to have adequate resources. The weekly scheduling of operations for chosen patients and the problem of assigning procedures to operate rooms in the event of ambiguity about surgery duration and the coming of emergency patients depending on a flexible policy (capacity reservation) were studied in this research. We have a list of chosen patients awaiting surgery and some surgeons with various specialties who should be booked in the event of ambiguity about the length of surgery and the advent of emergency patients on their surgeon's days off. The scheduling of operating room units and intensive care units is taken into account in this research. The problem under investigation has several restrictions. These considerations comprise the intensive care unit (ICU), the restricted time accessible for work, the noninterference of procedures involving an operating room, and the noninterference of operations involving a surgeon because most multiple ORs are outfitted with specialized equipment and can accommodate a variety of operations. We approached the operating room separately, and it is also conceivable to add a restricted number of beds to the intensive care units (ICUs) in the event of a bed constraint.

The article "Presented a Framework of Computational Modeling to Identify the Patient Admission Scheduling Problem in the Healthcare System" was published in 2022. Journal: J Healthc Eng.

The following are the assumption of the theory in question.

(i) All patients are operated, both nonpreferentially and selectively, in the many ORs available
(ii) The value of a weekly routine cannot be overstated
(iii) It is possible to schedule multiple rooms
(iv) The length of the operation varies
(v) Emergency patients are also admitted at random
(vi) The objectives of patients are taken into account while scheduling
(vii) It is feasible to do business outside of regular working hours (overtime)
(viii) Anesthesiologists, nurses, surgeons' assistants, and other human resources are available
(ix) Professionals, on the other hand, see constraints as the most valuable human resource
(x) The characteristics of operating rooms are the same
(xi) Index:
   
*p*: Set of all patients
   
*q*′: Set of all noninfectious patients
   
*p*′: Set of all nonemergency patients
   
*p*′: Set of all emergency patients
   
*o*: Set of all multiple ORs
   
*s*: A Set of all surgeons
   
*t*: A set of all available time blocks
   
*d*: Set of all available days
(xii) Parameters:
   
*C*_*pos*_: The expense of assigning the *P* th patient to the *O* th operating room and assigning the *s*  th surgeon to the *P* th patient
   
*D*_*p*′_: The expense of altering a nonemergency patient  *p*′s treatment plan
   
*EC*_*od*_: On the *d* th day, the expense of not utilizing the *o* operating room
   
*LC*_*od*_: On the *d* th day, the expense of excessive usage of the operating room
   
*δ*_*p*′_: The total number of modifications made to the nonemergency patient program *p*′ to this point
   
*U*_*d*_: Intensive care unit (ICU) shortfall cost per day *d*
   
*du*_*p*_: When the patient's *p* operation lasts, the number of blocks
   
*cl*_*q*_: After *q* th operation, the number of time blocks required to clean the operating area
   
*da*_*p*_: The most recent time frame (day) in which we are permitted to operate on my *p* th patient
   
*dI*_*p*_: The number of days in the intensive care unit that the *p* th patient should spend (ICUs)
   
*R*_*po*_: If the *p* th patient may be allocated to the *o* th operating room, *R*_*po*_ is one; otherwise, it is zero
   
*Q*_*ps*_: If the *p* th patient can be allocated to the *s* surgeon, *Q*_*ps*_ equals one; otherwise, it equals zero
   
*G*: The number of nonemergency surgical time blocks a surgeon can do each day
   
*HN*_*od*_: The number of time blocks allotted on the *d* th day to run the *o* th operating room
   
*HS*_*od*_: Max number of extra work block for chosen patients in the *o* operating room on the *d* th day
   
*HO*_*od*_: The maximum number of time blocks that emergency patients can utilize the operating room after the authorized time blocks linked to the *o* operating room on the *d* th day
   
${\tilde{HM}}_{od}$: The amount of time allotted to emergency patients in the *o* operating room on day *d*; this parameter has a usual distribution with $\;E\left({\tilde{HM}}_{od}\right)$ as the mean and $Var\left({\tilde{HM}}_{od}\right)$ as the variance
   
*MT*_*s*_^*max*^: The *s* physician is max working hours on the planning
   
${\tilde{WICU}}_{d}$: The number of intensive care unit (ICU) units allotted to emergency patients; this variable has a normal distribution with $E\left({\tilde{WICU}}_{d}\right)$ as the mean and $Var\left({\tilde{WICU}}_{d}\right)$ as the variance
   
${\tilde{Cicu}}_{d}$: The number of boards accessible in the intensive care unit (ICUs); this variable has a normal distribution with $E\left({\tilde{Cicu}}_{d}\right)$ as the mean and $\text{Var}\left({\tilde{\text{Cicu}}}_{d}\right)$ as the variance
   
*x*_*postd*_^0^: It is one if the *p* th patient's preoperative surgery in the operating room begins utilizing the *s* th surgeon in the *t*  th time block on the *d* th day; otherwise, it is zero
   
*θ*: The most significant number of times a nonemergency patient's treatment schedule can be altered
(xiii) Decision variables:
   
*x*_*postd*_: If the *p* th patient's operation is started in the operating room by the *s* th surgeon in the *t*  th time block on the dth day, *x*_*postd*_ is one; otherwise, it is zero
   
${\bar{x}}_{postd}$: If the *p* th patient's operation is done in the operating room by the *s* th surgeon in the *t*  th time block on the *d* th day, ${\bar{x}}_{postd}$ equals one; otherwise, it equals zero
   
*y*_*pd*_: If the *p* th patient is admitted to the intensive care unit (ICU) on the dth day, *y*_*pd*_ equals one; otherwise, it equals zero
   
${\bar{y}}_{pd}$: If the *p* patient is in the intensive care unit (ICUs) on the *d* th day, ${\bar{y}}_{pd}$ is one; otherwise, it is zero
   
*Z*_*d*_: The number of intensive care beds in limited supply on the *d* th day
   
*γ*_*p*′_: If the treatment plan for the *p*'th nonemergency patient is altered, *γ*_*p*′_ equals one; otherwise, it equals zero
   
*α*_*od*_: The length of time on the *d* th day that the operating room will not be used
   
*β*_*od*_: On the *d* th day, the amount of time to misuse the operation room
(xiv) Mathematical model.
(xv) This section contains a list of patients.
   
*p*: All patients, including patients, are gathered
   
*q*: Compile a list of all infected patients
   
*q*′: All noninfectious patients are gathered
   
*p*′: All nonemergency patients are gathered

This area does not have any emergency patients; only the capacity is set aside for them.

(5) $$\begin{array}{c} \text{Min}Z=\overset{P}{\underset{p=1}{\sum }}\overset{O}{\underset{o=1}{\sum }}\overset{S}{\underset{s=1}{\sum }}\overset{T}{\underset{t=1}{\sum }}\overset{D}{\underset{d=1}{\sum }}C_{pos}\times x_{postd}\;+\overset{O}{\underset{o=1}{\sum }}\overset{D}{\underset{d=1}{\sum }}EC_{od}\times \alpha_{od}+\overset{O}{\underset{o=1}{\sum }}\overset{D}{\underset{d=1}{\sum }}LC_{od}\times \beta_{od}+\overset{D}{\underset{d=1}{\sum }}U_{d}\times Z_{d\;}, \end{array}$$

(6) $$\begin{array}{c} \overset{O}{\underset{o=1}{\sum }}\overset{S}{\underset{s=1}{\sum }}\overset{T}{\underset{t=1}{\sum }}\overset{D}{\underset{d=1}{\sum }}x_{postd}=1\;\forall p\;, \end{array}$$

(7) $$\begin{array}{c} {\bar{x}}_{postd}=\overset{t}{\underset{t^{\prime }=\text{max}\left(t-du_{p}+1,1\right)}{\sum }}\begin{array}{c} x_{post^{\prime }d}\forall \;p,o,s,t,d\\ \; \end{array}, \end{array}$$

(8) $$\begin{array}{c} \overset{P}{\underset{\begin{array}{c} p=1\\ p\neq q \end{array}}{\sum }}\overset{S}{\underset{s=1}{\sum }}\overset{t^{\prime }+du_{q}+cl_{q}-1}{\underset{t=t^{\prime }}{\sum }}x_{postd}\leq 1-\overset{S}{\underset{s=1}{\sum }}x_{qost^{\prime }d}\;\forall \;q,o,t^{\prime },d\;, \end{array}$$

(9) $$\begin{array}{c} \overset{P}{\underset{p=1}{\sum }}\overset{S}{\underset{s=1}{\sum }}{\bar{x}}_{postd}\leq 1\forall \;o,t,d\;, \end{array}$$

(10) $$\begin{array}{c} \overset{P}{\underset{p=1}{\sum }}\overset{O}{\underset{o=1}{\sum }}{\bar{x}}_{postd}\leq 1\forall s,t,d\;, \end{array}$$

(11) $$\begin{array}{c} \overset{P}{\underset{p=1}{\sum }}\overset{O}{\underset{o=1}{\sum }}\overset{S}{\underset{s=1}{\sum }}\overset{T}{\underset{t=1}{\sum }}\overset{D}{\underset{d=da_{p}+1}{\sum }}x_{postd}=0, \end{array}$$

(12) $$\begin{array}{c} \overset{S}{\underset{s=1}{\sum }}\overset{T}{\underset{t=1}{\sum }}\overset{D}{\underset{d=1}{\sum }}x_{postd}\leq R_{po\;}\forall p,o, \end{array}$$

(13) $$\begin{array}{c} \overset{O}{\underset{o=1}{\sum }}\overset{T}{\underset{t=1}{\sum }}\overset{D}{\underset{d=1}{\sum }}x_{postd}\leq Q_{ps}\forall p,s\;, \end{array}$$

(14) $$\begin{array}{c} \overset{P^{\prime }}{\underset{p^{\prime }=1}{\sum }}\overset{O}{\underset{o=1}{\sum }}\overset{T}{\underset{t=1}{\sum }}{\bar{x}}_{p^{\prime }ostd}\leq G\;\forall s,d\;, \end{array}$$

(15) $$\begin{array}{c} \overset{P^{\prime }}{\underset{p^{\prime }=1}{\sum }}\overset{S}{\underset{s=1}{\sum }}\overset{T}{\underset{t=1}{\sum }}{\bar{x}}_{p^{\prime }ostd}\leq HN_{od}+HS_{od}\forall \;o,d\;, \end{array}$$

(16) $$\begin{array}{c} \overset{P^{\prime }}{\underset{p^{\prime }=1}{\sum }}\overset{S}{\underset{s=1}{\sum }}\overset{T}{\underset{t=1}{\sum }}{\bar{x}}_{p^{\prime }ostd}+{\tilde{HM}}_{od}\leq HN_{od}+HO_{od\;}\forall \;o,d, \end{array}$$

(17) $$\begin{array}{c} \alpha_{od}\geq HN_{od}-\overset{P}{\underset{p=1}{\sum }}\overset{S}{\underset{s=1}{\sum }}\overset{T}{\underset{t=1}{\sum }}{\bar{x}}_{postd}\forall o,d\;, \end{array}$$

(18) $$\begin{array}{c} \beta_{od}\geq \overset{P^{\prime }}{\underset{p^{\prime }=1}{\sum }}\overset{S}{\underset{s=1}{\sum }}\overset{T}{\underset{t=1}{\sum }}{\bar{x}}_{postd}-HN_{od\;}\forall o,d, \end{array}$$

(19) $$\begin{array}{c} \overset{P^{\prime }}{\underset{p^{\prime }=1}{\sum }}\overset{O}{\underset{o=1}{\sum }}\overset{T}{\underset{t=1}{\sum }}\overset{D}{\underset{d=1}{\sum }}{\bar{x}}_{p^{\prime }ostd}\leq MT_{s}^{max}\forall \;s,d, \end{array}$$

(20) $$\begin{array}{c} \overset{O}{\underset{o=1}{\sum }}\overset{S}{\underset{s=1}{\sum }}\overset{T}{\underset{t=1}{\sum }}{\bar{x}}_{postd}\leq M\times y_{pd\;}\forall p,d, \end{array}$$

(21) $$\begin{array}{c} {\bar{y}}_{p\;d}=\overset{d}{\underset{d^{\prime }=\text{max}\left(d-dI_{p}+1,1\right)}{\sum }}y_{pd^{\prime }}\forall p,d, \end{array}$$

(22) $$\begin{array}{c} \overset{P^{\prime }}{\underset{p^{\prime }=1}{\sum }}{\bar{y}}_{p^{\prime }d}+{\tilde{WICU}}_{d}\leq {\tilde{Cicu}}_{d}+Z_{d\;}\forall \;d, \end{array}$$

(23) $$\begin{array}{c} 1-\overset{Q^{\prime }}{\underset{q^{\prime }=1}{\sum }}\overset{S}{\underset{s=1}{\sum }}\overset{T}{\underset{t=t^{\prime }+1}{\sum }}x_{q^{\prime }ostd}\geq \overset{S}{\underset{s=1}{\sum }}x_{qost^{\prime }d\;}\forall \;q,o,t^{\prime },d. \end{array}$$

Equation (5)'s goal is to reduce the expense of assigning patients to many ORs and surgeons, not utilizing and overusing multiple ORs, and the cost of overusing an intensive care unit. Restriction (6) guarantees that each patient (including emergency and nonemergency) is allocated to a particular operating room and surgeon on a given day and for a specific amount of time. Restriction (7) guarantees that each patient receives the appropriate time blocks for time block surgery. Limit (8) guarantees that each operating room is cleaned after surgery for each contaminated patient for at least *cl*_*q*_  minutes. Limit (9) indicates that each operating room can only execute one surgery during each time block in a day. Restriction (10) specifies that each surgeon can only do one surgery in one operating room during each time block in a day. Restriction (11) guarantees that each patient is allocated to a specific operating room and surgeon before a deadline. Restrictions (12) and (13) guarantee that each patient is allocated to a particular operating room and surgeon. Restriction (14) guarantees that physicians do not work more than a specific number of hours per day on nonemergency patients. Patients can utilize each operating room as much as they like in emergency and nonemergency situations, according to restrictions (15) and (16). Restrictions (17) and (18) measure the amount of time that operating rooms are overused and underutilized for nonemergency patients on various days. The restriction (19) is linked to surgeons' maximum working hours. It regulates the amount of time on nonemergency patients. Restriction (20) guarantees that each patient who has surgery is admitted to the critical care unit. The restriction above (21) guarantees that each patient receives a bed in an intensive care unit (ICU) for the number of days necessary for admission. Restriction (22) estimates the number of bed limitations for emergency and nonemergency patients based on the intensive care unit's capacity. Daily, restriction (23) guarantees that infected patients are the last patients allocated to operating rooms.

The article "Presented a Framework of Computational Modeling to Identify the Patient Admission Scheduling Problem in the Healthcare System" was published in 2022. Journal: J Healthc Eng.

## 4. Computational Results

A small-scale instance is presented for each suggested model in this part to comprehend and verify the concepts above. In the first half of the instance, there are three operating rooms and three surgeons. Each day is separated into six time periods. Ten patients were scheduled in different operating rooms and intensive care units, comprising eight chosen patients and three infectious patients (patients 1, 2, and 3). The number of time intervals permitted to work for each room each day *HN*_*od*_  is different in this case. Over time, it is deemed if the patient's room allotment exceeds this amount (see Figures 4–7).

The results are derived from the GAMS program output (see Figures 8–10).

## 5. Discussion

Compared to other sectors, healthcare quality assessment is doubly important due to the sensitivity of the services provided in this area on the one hand due to their relationship with death and life of individuals and on the other hand due to the asymmetry of information between providers and patients. Along with reducing the length of hospital stays, improving the quality of healthcare can also reduce mortality. Healthcare system managers can identify their opportunities and weaknesses with a tool that measures patient expectations and perceptions. A manager who identifies and covers service quality gaps will likely increase customer satisfaction by increasing customer perception of service quality. From the point of view of outpatients, not all aspects of service quality were in good condition. This indicates a gap between the expectations and perceptions of clients of the quality of services provided in this center, which needs to be improved in all its dimensions. For this reason, it is suggested that managers pay more attention to patients' needs and provide appropriate services to reduce the existing quality gap. Trying to reduce the gap between patients' expectations and perceptions will lead to greater satisfaction and ultimately loyalty and return to the organization. Also, by using the SERVQUAL model (as one of the quality measurement tools), managers are able to evaluate the quality of services from the perspective of patients as the most important customers, and with proper planning and correction of existing disorders and weaknesses, ultimately improved service quality is possible. Based on the literature review described above, the performance of outpatient facilities in the different departments evaluated in the healthcare clinic has greatly improved. To improve the efficiency of outpatient care, various techniques such as scheduling, modeling, and artificial intelligence are used to create a patient-centered appointment cycle. Treatment duration varies greatly depending on the patient. The challenge is choosing which model is more effective despite the fact that we have studied several articles and shown the benefits of several models. Since many scientists in this field have conducted simulation work, we can conclude that separate event simulation offers the most advantages and a better understanding of how to overcome the restrictions. In general, discrete-event simulation is an effective method of coordinating the many scheduling techniques required for healthcare. It also has a larger scale than classical Markov chain optimization, which makes it perfect for this application. It is imperative that our industry meet the rigorous design criteria that decision-makers will accept because the dangers are minimal and straightforward.

The article "Presented a Framework of Computational Modeling to Identify the Patient Admission Scheduling Problem in the Healthcare System" was published in 2022. Journal: J Healthc Eng.

## 6. Conclusion and Limitation

Healthcare in the United States is complicated and expensive. Therefore, there are many opportunities for researchers from a variety of disciplines to contribute to the improvement of healthcare systems. A hospital's operating room (OR) generates the most income and expense, according to healthcare analysts. In this study, we looked at existing modeling techniques for outpatient appointment scheduling in the healthcare industry. More than 200 publications are examined in this respect better to understand outpatient appointment scheduling issues in the literature. Researchers have paid great attention to the scheduling issue in the twenty-first century. Published technical OR scheduling publications have steadily increased since 2000. Rather than that, it reflects the diversity of viewpoints and healthcare contexts around the world on the issue. The reader may see an increasing trend of study interest in recent years (Figure 1) due to expanded hospital resources based on the data reports provided in this research. Despite the abundance of literature on outpatient appointment scheduling, there are several ways to enhance the current research, such as establishing planning models, performance metrics, and forecasting skills under various generalized situations. More research, for example, may be designed to focus on developing timetables that can be performed successfully on this issue.

It may be possible to create alternative healthcare access solutions by understanding scheduling systems' performance dynamics. It is necessary to have a different area of inspection in order to reduce overbooking. Healthcare access and service delivery will likely be scrutinized more closely by the general public due to their desire to improve. Mathematics can also be used to model numerous providers, such as double bookings, overtime expenses, and increasing the effectiveness time of visiting doctors. A mathematical model for the patient admission scheduling problem with stochastic arrivals and departures is the subject of this study. We discuss how we can apply our model to real-world problems. We present a solution technique for efficient computing, a numerical model analysis, and examples to demonstrate the method. In this study, we examined the challenge of assigning procedures to operating rooms in the face of ambiguity regarding surgery length and emergency arrivals based on a flexible policy (capacity reservations). Using simple numerical examples, we demonstrate that the proposed methods derived from deterministic models are inadequate compared to the answers obtained from our stochastic model. Similarly, we use heuristics to estimate the objective function to build more complicated numerical examples for large-scale issues, showing that our methodology can be applied quickly to real-world situations. [30, 77].

The article "Presented a Framework of Computational Modeling to Identify the Patient Admission Scheduling Problem in the Healthcare System" was published in 2022. Journal: J Healthc Eng.

### 6.1. Future Work

Researchers should examine how outpatients and walk-ins unexpectedly arrive at clinics, disrupting operations. A discrete-event simulation technique is often used in healthcare for real-time decision-making but is rarely discussed publicly. In healthcare applications, such as screening and illness management, discrete-event simulation is the most accurate modeling method. Let's use a version of healthcare optimization. In such a case, different patients must be convinced of their benefits and limitations within the healthcare industry. Further studies are needed to evaluate how walk-in outpatients affect the timeliness of scheduled arrivals in greater detail. A further area of future investigation would be the formulation of sequencing issues based on individual unpunctuality habits. A game theory approach could be used to extend current models to account for physicians, nurses, and patients' unpredictable behavior. As a research gap, scheduling difficulties during outpatient appointments might be used to simulate the multistage health process, like the initial examination, drug test, and preparation of patients, or to optimize multivisit schedules in clinics.

## Figures and Tables

**Figure 1:** Number of the covered article.

**Figure 2:** Scheduling appointments and allocating resources integrated [24].

**Figure 3:** The pie chart for the applications to patient and outpatient scheduling problems.

**Figure 4:** The amount of time allowed to work for room 1 and each day.

**Figure 5:** The amount of time allowed to work for room 2 and each day.

**Figure 6:** The amount of time allowed to work for room 3 and each day.

**Figure 7:** Intensive care schedule (part 1).

**Figure 8:** The amount of time not to use the operating room 1.

**Figure 9:** The amount of time not to use the operating room 2.

**Figure 10:** The amount of time not to use the operating room 3.

**Table 1:** Healthcare scheduling in optimization context: a review.

References	Method	Uncertain/elective
[56]	Programming in a stochastic manner	Uncertainty
[46]	Programs that use integers	—
[57]	Linear stochastic program	Uncertainty
[58]	Exact solution algorithm based on branch and price	
[59]	Algorithm of branching and bounding	—
[60]	Local search and heuristics	Elective
[61]	Dynamic stochastic programming	Elective
[62]	Light robustness approach and mixed-integer linear formulation	Elective
[63]	Model of integer linear programming	Elective
[64]	Model of stochastic dynamic programming	Elective
[65]	Bi-criteria heuristics discrete-event simulation model heuristics GA	Elective
[66]	Binary programming, local search, integer programming	Elective/emergency
[67]	Discrete-event model	Uncertain
[68]	Discrete event dynamic system	Elective

The article "Presented a Framework of Computational Modeling to Identify the Patient Admission Scheduling Problem in the Healthcare System" was published in 2022. Journal: J Healthc Eng.

**Table 2:** Calculation of the objective function.

The value of the objective function	Solving time (seconds)
3569	0.0085

## Data Availability

Data are available and can be provided over the emails querying directly to the corresponding author (mohsenasghari1990@ut.ac.ir).
